RETRACTED

# Study on the Effect of Different Doses of Hydromorphone on the Time Response and Postoperative Analgesia of Ropivacaine in Ultrasound-Guided Suprailiac Fascia Inguinal Block

**DOI:** 10.1155/2021/9691062

**Published:** 2021-10-14

**Authors:** Baiyun Wang, Bingbing Hu, Huanhui Zhong, Chengda Zhao

**Affiliations:** The Affiliated Nanhua Hospital, Department of Anesthesiology, Hengyang Medical College, University of South China, Hengyang 421001, Hunan, China

## Abstract

**Objective:**

To investigate the effects of different doses of hydromorphone under the guidance of ultrasound on ropivacaine blocking the superior inguinal iliac fascia and postoperative analgesia.

**Methods:**

From January 2020 to June 2021, 90 American Society of Anesthesiologists (ASA) I-II patients undergoing elective total hip arthroplasty (THA) were selected and randomly divided into 3 groups, 30 patients in each one. Ultrasound-guided superior inguinal iliac fascia block was performed in the patients of the 3 groups before operation. The L group: 0.3% ropivacaine 30 ml; the H1 group: 0.3% ropivacaine + 25 *μ*g/kg hydromorphone 30 ml; the H2 group: 0.3% ropivacaine + 50 *μ*g/kg hydromorphone 30 ml. The time until the occurrence of pain, pain intensity, sufentanil remedial dose, the number of PCIA presses, and effective times were compared among the 3 groups. The VAS and Ramsay scores of 3 groups were recorded at 12 h, 24 h, 36 h, and 48 h after operation.

**Results:**

The time from the end of surgery to the appearance of pain in the H2 group was higher than that in the H1 group and the L group, and the time in the H1 group was higher than that in the L group (*P* < 0.05). The VAS score in the H2 group was lower than that in the H1 group and the L group, and the VAS score in the H1 group was lower than that in the L group (*P* < 0.05). The VAS scores of 12 h, 24 h, 36 h, and 48 h after operation in the H2 group were lower than those of the H1 group and the L group, and the H1 group was lower than the L group (*P* < 0.05). The Ramsay scores at 12 h, 24 h, 36 h, and 48 h after operation in the H2 group and the H1 group were higher than those in the L group (*P* < 0.05), and the difference was not statistically significant in the H2 group and the H1 group (*P* > 0.05). The remedial dosage of sufentanil, times of PCIA compression, and effective times in the H2 group were lower than those in the H1 group and the L group, and the level in the H1 group was lower than that in the L group (*P* < 0.05). The incidence rates of adverse reactions in the L group, the H1 group, and the H2 group were 13.33%, 23.33%, and 30.00%, respectively. There was no significant difference in the incidence rate of adverse reactions among the 3 groups (*P* > 0.05).

RETRACTED

**Conclusion:**

25 *μ*g/kg and 50 *μ*g/kg hydromorphone used in the ultrasound-guided superior inguinal iliac fascia block can enhance the time effect of ropivacaine and improve analgesic effects, with good safety. In addition, time effect and analgesic effect of 50 *μ*g/kg hydromorphone in enhancing ropivacaine were more obvious.

## 1. Introduction

With the aging of the population and the increase of car accidents and trauma, the rate of hip degeneration and fracture increases year by year [1, 2]. Total hip arthroplasty (THA) is the most effective treatment for hip degeneration and fracture. Post-THA patients have severe trauma and pain. At the same time, these patients often suffer from chronic diseases such as hypertension and diabetes and are prone to postoperative complications such as pulmonary infection and cardiovascular and cerebrovascular accidents. Studies have shown that ultrasound-guided superior inguinal iliac fascial block used after THA can relieve postoperative pain and reduce the incidence of complications [3]. However, the block time of single inguinal suprailiac fascia is limited, and severe reflex pain is easy to occur after symptoms subside. Ultrasound-guided continuous iliac fascia block can solve the pain, and the block time is short, and it can bounce back. However, continuous catheterization may lead to infection, catheter removal, and other risks. Therefore, exploring how to prolong the duration of a single nerve block and enhance its effect has become a hot topic. Hydromorphone can prolong the acting time of the abdominal transverse fascia and enhance the acting effect. Hydromorphone exerts the analgesic effect by exciting the *μ*-receptor and is widely used for clinical analgesia because of its low incidence of adverse reactions such as skin pruritus and respiratory depression [4–6]. Hydromorphone combined with local anesthetics can significantly prolong the analgesic effect when used in the block of the upper iliac fascia in the groin. However, the appropriate dose of hydromorphone combined with ropivacaine for superior inguinal iliac fascia block is still unclear. This study explored the effects of different concentrations of hydromorphone on the ropivacaine time and postoperative analgesia in ultrasound-guided superior inguinal iliac fascia block for THA patients, so as to provide clinical reference for the appropriate dose of hydromorphone combined with ropivacaine for THA patients. Now, we report the following.

## 2. Data and Methods

### 2.1. General Information

The informed consent form was signed by the patients and their families with the approval of the Hospital Ethics Committee. A total of 90 American Society of Anesthesiologists (ASA) I-II patients undergoing elective THA in our hospital from January 2020 to June 2021 were selected and randomly divided into 3 groups, 30 patients in each group. Ultrasound-guided superior inguinal iliac fascia block was performed in the patients of the 3 groups before operation. The L group: 0.3% ropivacaine 30 ml; the H1 group: 0.3% ropivacaine + 25 *μ*g/kg hydromorphone 30 ml; the H2 group: 0.3% ropivacaine + 50 *μ*g/kg hydromorphone 30 ml. The inclusion criteria were as follows: patients meeting the indication of THA surgery; there was no allergic reaction or contraindication to the narcotic drugs to be used in this study; patients were in good mental condition and can cooperate with the implementation of the treatment process. The exclusion criteria were as follows: coagulation disorders; suffering from peripheral nerve disease; suffering from mental diseases; suffering from serious cardiovascular and cerebrovascular diseases, diabetes, and other complications; infection at the puncture site; ropivacaine and hydromorphone allergy; who cannot cooperate.

RETRACTED

### 2.2. Research Methods

All patients were deprived of food and water for 6 h. After entering the operating room, intravenous access was opened to monitor ECG, oxygen saturation, blood pressure, and respiration, and oxygen was inhaled through the conventional nasal catheter (2 L/min). Ultrasound-guided groin superior iliac fascia block was performed in both groups. The “hillside sign” was adopted for positioning. The patients were recumbent, and the high-frequency probe was taken. The probe was placed at the position of the anterior superior iliac spine. The direction of the probe was towards the navel to identify the anterior superior iliac spine, iliopsoas muscle on the surface of the ilium, and iliac fascia with high echo on the surface of the iliopsoas muscle. The ultrasonic images were like “hillside” from superficial to deep, including subcutaneous fat, external oblique muscle or aponeurosis, internal oblique muscle, transverse muscle, iliopsoas muscle, and ilium. Precise puncture was performed under the guidance of ultrasound. The needle was inserted in the plane, and it was withdrawn while being inserted. The tissue was separated using the water separation technology, and the drug was injected between the iliopsoas muscle and iliac fascia. Patients in the *L* group were diluted to 30 ml with 90 mg ropivacaine + normal saline in the iliac fascia space. Patients in the H1 group were diluted to 30 ml with 90 mg ropivacaine + 25 *μ*g/kg hydromorphone + normal saline in the iliac fascia space. Patients in the H2 group were diluted to 30 ml with 90 mg ropivacaine + 50 *μ*g/kg hydromorphone + normal saline in the iliac fascia space. After the effectiveness of the block was confirmed, a single spinal anesthesia was performed in the lumbar intervertebral space 2-3. A single dose of 1 ml of 10% glucose plus 1% 2 ml of ropivacaine mixture (2.5 ml) was administered, and the patient was kept in the supine position with the control plane from T8 to T10.

RETRACTED

Patient-controlled analgesia (PCIA) was performed in 3 groups after operation. PCIA formula is sufentanil 2 ug/kg + ondansetron 8 mg + normal saline which were diluted to 100 ml, and the parameters were set as 2 ml/h, locked for 10 min, and added 2 ml/time. The patient was asked to call the Department of Anesthesiology if he/she suffers from pain (resting VAS score ≥3 points). At the same time, the patient's VAS score is evaluated by phone. The anesthesiologist arrives at the ward within 15 min, reassesses the VAS score, starts PCIA at the same time, and carries out an additional observation. The patient is observed for 10 min. If the patient's VAS score is ≤3 points, no treatment is required. If the VAS score >3 points, continue to add until the VAS score ≤3 points.

The time until the occurrence of pain, pain intensity, sufentanil remedial dose, the number of PCIA presses, and effective times were compared among the 3 groups. The VAS and Ramsay scores at 12 h, 24 h, 36 h, and 48 h after operation in the 3 groups were recorded.

### 2.3. Statistical Methods

SPSS 20.0 software was used for processing. The measurement data of the experimental data were expressed as mean ± standard deviation, and the *t*-test was used for pairwise comparison. One-way analysis of variance was used for comparison among groups, and repeated measures were used for comparison among groups at the same time point, and the analysis of variance was used for multigroup comparison. The count data were expressed as rate, and the comparison was performed using the chi-square test. The test level was *α* = 0.05, and *P* < 0.05 indicated that the difference was statistically significant.

## 3. Results

### 3.1. Comparison of General Information and Operation Time Comparison among the Three Groups

There were no significant differences in gender, age, body weight, ASA grade, or operation time among the three groups (*P* > 0.05), as shown in Table 1.

### 3.2. Comparison of Time to Onset of Pain and Pain Intensity among the Three Groups of Patients

The differences in the time to the occurrence of pain and the pain intensity among the three groups were statistically significant (*P* < 0.05). The time from the end of surgery to the appearance of pain in the H2 group was higher than that in the H1 group and the L group, and the time in the H1 group was higher than that in the L group (*P* < 0.05). The VAS scores of the H2 group were lower than those of the H1 group and the L group, and the VAS score of the H1 group was lower than that of the L group (*P* < 0.05), as shown in Figure 1.

RETRACTED

### 3.3. Comparison of the VAS Scores at 12 h, 24 h, 36 h, and 48 h after Operation among the Three Groups

The VAS scores of the patients in the three groups gradually increased at 12 h and 24 h after operation and reached the highest at 36 h after operation, while the VAS score of 48 h after operation decreased. The VAS scores of the H2 group at 12 h, 24 h, 36 h, and 48 h after operation were lower than those of the H1 group and the L group, and the H1 group was lower than the L group, and the differences were statistically significant (*P* < 0.05), as shown in Figure 2.

### 3.4. Comparison of the Ramsay Scores at 12 h, 24 h, 36 h, and 48 h after Operation among the Three Groups

There were no significant changes in the Ramsay scores of 12 h, 24 h, 36 h, and 48 h after operation in the three groups. The Ramsay scores at 12 h, 24 h, 36 h, and 48 h after operation in the H2 group and the H1 group were higher than those in the L group (*P* < 0.05), and the difference was not statistically significant in the H2 group and the H1 group (*P* > 0.05), as shown in Figure 3.

### 3.5. Comparison of Postoperative Sufentanil Remedial Dose, PCIA Compression Times, and Effective Times among the Three Groups of Patients

The remedial dosage of sufentanil, times of PCIA compression, and effective times in the H2 group were lower than those in the H1 group and the L group, and the level in the H1 group was lower than that in the L group. The differences were statistically significant (*P* < 0.05), as shown in Figure 4.

### 3.6. Comparison of the Incidence of Adverse Reactions among the Three Groups

The incidence rates of adverse reactions in the L group, the H1 group, and the H2 group were 13.33%, 23.33%, and 30.00%, respectively. There was no significant difference in the incidence rate of adverse reactions among the three groups (*P* > 0.05), as shown in Figure 5.

## 4. Discussion

Postoperative pain is acute pain that often leads to poor emotional response. In particular, it increases the risk of organ dysfunction, prolongs hospital stay, delays recovery, and increases the incidence of readmission [7]. Post-THA pain was mainly caused by capsular pain in the hip and pain in the surgical incision, which was innervated by the main femoral joint branches and the lateral femoral cutaneous nerve. Studies have shown that superior inguinal iliac fascia block can well block the femoral nerve and the lateral femoral cutaneous nerve [8]. At present, there are many approaches to block the superior inguinal iliac fascia, and the experimental group chose the “hillside sign” approach for block. Bullock et al.'s study and other studies show that the improved superior inguinal iliac fascia block can accurately block the lateral femoral cutaneous nerve and provide good analgesia for patients [9]. Superior inguinal iliac fascia block has the risk of perforating the abdominal cavity and damaging blood vessels and nerves. Therefore, ultrasound-guided puncture is often performed clinically.

RETRACTED

Ropivacaine is widely used for nerve block due to its high safety and good analgesic effect. Opioids have been used as adjuvants of local anesthetics for many years, and many studies have shown that the combination of opioids and local anesthetics can enhance the synergistic effect of the two and prolong the action time of the drugs [10, 11]. In view of the strong respiratory inhibition by morphine and the possibility that the metabolite morphine-6-gluconic acid may aggravate the renal burden of patients and increase the incidence of drowsiness and nausea, morphine has limited its application in the peripheral nerve block due to severe opioid adverse reactions [12]. Hydromorphone, a pure *μ*-receptor agonist, a derivative of morphine, has been widely used for perioperative analgesia due to its good analgesic effect and less adverse reactions. More and more studies have shown that hydromorphone can prolong the time-effect limit of the ropivacaine nerve block. However, when ropivacaine is used for the iliofascial block, there are few reports about the effect of hydromorphone with proper concentration on its time-effect limitation [13].

In this study, 25 *μ*g/kg and 50 *μ*g/kg hydromorphone were selected for use in patients with THA at a dose within the effective range. The results showed that the time from the end of surgery to onset of pain in the H2 group was higher than that in the H1 group and the L group, and the time in the H1 group was higher than that in the L group. Moreover, the pain scores in the H2 group were lower than those in the H1 group and the L group, and the pain score in the H1 group was lower than that in the L group. These results indicated that the addition of 50 *μ*g/kg hydromorphone to 0.3% ropivacaine for superior inguinal iliac fascia block could prolong the action time of ropivacaine, and the addition of 50 *μ*g/kg hydromorphone had a more significant effect in prolonging the action time of ropivacaine. The results also showed that the VAS scores of the three groups increased gradually at 12 h and 24 h after operation, reached the highest at 36 h after operation, and decreased at 48 h after operation. The VAS scores of the H2 group at 12 h, 24 h, 36 h, and 48 h after operation were lower than those of the H1 group and the L group, and the H1 group was lower than the L group. The Ramsay scores of patients in the three groups increased gradually at 12 h, 24 h, 36 h, and 48 h after operation. The Ramsay scores at 12 h, 24 h, 36 h, and 48 h after operation in the H2 group and the H1 group were higher than those in the L group, and there was no significant difference between the H2 group and the H1 group. The results showed that, with the increase of hydromorphone dose, the postoperative analgesia effect of patients was significantly improved [14–16].

RETRACTED

Sufentanil is an opioid analgesic, which takes effect quickly, but it is easy to produce adverse reactions such as nausea and vomiting, and it is easy to cause oversedation, which has a negative impact on patients' early getting out of bed activities [17]. The results of this study showed that the remedial dosage of sufentanil, the number of PCIA presses, and the effective times in the H2 group were lower than those in the H1 group and the L group, and the number in the H1 group was lower than that in the L group. These results indicated that higher concentration of hydromorphone combined with ropivacaine could significantly reduce the dosage of sufentanil and avoid the excessive sedative effect of large doses of analgesic drugs, which affected postoperative rehabilitation. The mechanism may be related to the fact that hydromorphone prolongs the analgesic time of patients and reduces postoperative stress response [18, 19]. The results also showed that there was no significant difference in the incidence of adverse reactions between the three groups. It may be related to the reduction of sufentanil dosage and the incidence of postoperative adverse reactions in the hydromorphone group, and it is also beneficial to improve the quality of postoperative recovery [20].

In this study, the relatively long interval in pain assessment eliminated the fatigue score of patients and improved the accuracy of assessment. However, there are still some shortcomings in this study, for example, the sample size was small and the blood concentration of hydromorphone due to limited conditions. In the future work, we should cumulatively increase the sample size and determine the blood concentration of hydromorphone to further explore the specific mechanism.

## 5. Conclusion

In summary, the applications of 25 *μ*g/kg and 50 *μ*g/kg hydromorphone in ultrasound-guided superior inguinal iliac fascia block can both enhance the time effect of ropivacaine and enhance analgesic effects with good safety. In addition, time effect and analgesic effect of 50 *μ*g/kg hydromorphone in enhancing ropivacaine were more obvious.

RETRACTED

## Figures and Tables

**Figure 1:** General information and operation time comparison among the three groups. Note: compared with the L group, ^*∗*^*P* < 0.05. Compared with the H1 group, ^#^*P* < 0.05.

**Figure 2:** The VAS scores at 12 h, 24 h, 36 h, and 48 h after operation among the three groups. Note: compared with the L group, ^*∗*^*P* < 0.05. Compared with the H1 group, ^#^*P* < 0.05.

**Figure 3:** The Ramsay scores at 12 h, 24 h, 36 h, and 48 h after operation among the three groups. Note: compared with the L group, ^*∗*^*P* < 0.05.

**Figure 4:** Postoperative sufentanil remedial dose, PCIA compression times, and effective times among the three groups of patients. Note: compared with the L group, ^*∗*^*P* < 0.05. Compared with the H1 group, ^#^*P* < 0.05.

**Figure 5:** The incidence of adverse reactions among the three groups.

**Table 1:** General data and operation time of three groups of patients (%, $\bar{x}$ ± *s*).

Group	*n*	Male/female	Age (years)	Body weight (kg)	ASA I/II	Operation time (min)
L group	30	16/14	70.21 ± 7.12	56.13 ± 8.35	12/18	60.23 ± 9.47
H1 group	30	19/11	68.43 ± 8.24	54.45 ± 7.26	14/16	62.12 ± 8.35
H2 group	30	17/13	69.05 ± 8.05	54.92 ± 7.74	13/17	60.52 ± 8.37
*F* value		0.638	0.401	0.371	0.271	0.406
*P* value		0.727	0.671	0.691	0.873	0.667

## Data Availability

The data used to support the findings of this study are available from the corresponding author upon request.
